The article "Therapeutic Effect and Mechanism of Cinnamyl Alcohol on Myocardial Ischemia-Reperfusion Injury" was retracted in 2023. Reasons: signs of a paper mill; compromised peer review; unreliable results or conclusions.

# Therapeutic Effect and Mechanism of Cinnamyl Alcohol on Myocardial Ischemia-Reperfusion Injury

**DOI:** 10.1155/2022/5107948

**Published:** 2022-05-31

**Authors:** Hua Zhang, Jian Ye, Xu Wang, zongjun liu, Tao Chen, Junqing Gao

**Affiliations:** Department of Cardiology, Putuo Hospital, Shanghai University of Traditional Chinese Medicine, Shanghai 200062, China

## Abstract

**Objective:**

To investigate the effect of CA on autophagy and its molecular mechanism after myocardial ischemia/reperfusion injury (MI/RI).

**Methods:**

The MI/RI model was established by the ligation of the left anterior descending coronary artery with ischemia and reperfusion. *In vitro* cell models were established using hypoxia/reoxygenation. Western blot was used to determine the expression levels of beclin-1, P62, and LC3 II. The expression levels of IL-1*β*, IL-6, TNF*α*, and apoptosis-related genes Bax, Cyt-c, and Bcl-2 were detected by qRT-PCR. Cell activity was detected by CCK-8. Apoptosis was detected by TUNEL staining.

**Results:**

Beclin-1, P62, and LC3 II protein expression and LC3 II/LC3 I level were significantly increased after myocardial ischemia-reperfusion injury. Compared with model group, CA downregulated beclin-1, P62, and LC3 II protein expression and LC3 II/LC3 I level in the myocardium. The results of cell-level experiments showed that CA inhibited the autophagy response of the cardiomyocytes induced by hypoxia-reperfusion injury. Mechanism studies showed that CA targeted the inhibition of ATG12. Knocking down ATG12 reduces the production of inflammatory cytokines induced by H/R. The knockdown of ATG12 also reduced apoptosis and injury of the myocardial cells.

**Conclusion:**

Myocardial ischemia-reperfusion can enhance autophagy response and promote apoptosis. CA plays a protective role in myocardium by targeting ATG12, thereby inhibiting autophagy and improving myocardial cell apoptosis.

## 1. Introduction

MIRI is an inevitable process of myocardial injury in the clinical treatment of myocardial ischemia and recovery of myocardial blood supply, and its mechanism is very complex [1–3]. Studies have found that autophagy, a different endogenous protective mechanism related to apoptosis, is closely related to MIRI and has become a new therapeutic target for MIRI [4, 5]. Autophagy is a kind of cell autophagy phenomenon widely existing in eukaryotic organisms [6]. Under normal physiological conditions, autophagy can remove senescent organelles and degrade abnormally accumulated proteins, thus maintaining the stability of the body's internal environment [7]. When hypoxia or nutrient deficiency occurs, autophagy can degrade intracellular substances to produce amino acids and fatty acids to provide energy for the body and promote the synthesis of proteins and organelles [8]. Many pieces of evidence suggest that autophagy is involved in myocardial ischemia/reperfusion injury (MI/RI) and plays an important role in the pathological process of MI/RI [9, 10].

The article "Therapeutic Effect and Mechanism of Cinnamyl Alcohol on Myocardial Ischemia-Reperfusion Injury" was retracted in 2023. Reasons: signs of a paper mill; compromised peer review; unreliable results or conclusions.

ATG12, also known as autophagy associated protein 12, is a protein encoded by the ATG12 gene. ATG12 is an important protein associated with autophagy and apoptosis [11]. ATG12 is a human homologue of yeast proteins involved in autophagy. ATG12 and ATG5 form covalent connections through a ubiquitin-like conjugation system. The ATG12-ATG5 complex can further promote the binding of ATG8 to the lipid phosphatidylethanolamine and participate in the regulation of autophagy [12].

In recent years, studies on the regulation of MI/R injury using Traditional Chinese medicine from the perspective of the mitochondria have gradually increased, and it has shown good effects in improving MI/RI [13, 14]. More attention has been paid to the mechanism of inflammation and mitochondrial autophagy [15]. CA is the dried bark of *Cinnamomum cassia* Presl [16]. The main active ingredient of cinnamon is cinnamon oil [17]. As an important fine chemical intermediate, CA is widely used in the synthesis of essence, cosmetics, and medicine. However, whether CA can protect myocardial ischemia-reperfusion injury and its molecular mechanism have not been reported.

To explore the mechanism of autophagy regulation during myocardial ischemia-reperfusion injury is of great theoretical significance for future clinical interventions. In this study, we investigated whether CA could inhibit autophagy by inhibiting autophagy-related protein-12 (ATG12) and play a protective role in the myocardium. This study may provide a reliable experimental basis for the prevention and treatment of myocardial ischemia-reperfusion injury.

## 2. Methods

### 2.1. Animal Model of Myocardial Ischemia-Reperfusion Injury

Animals were purchased from Charles River Laboratory Animal Technology Co., LTD (Beijing, China). The laboratory maintains a constant temperature. Use disposable sawdust bedding material, and provide special drinking water and ordinary pellet feed for animals. The experiment was performed after 5 days of adaptive feeding. 30 SD rats were divided into sham operation group, model group, and CA intervention group by a random number table. The rats were fasting 12 hours before surgery and could not restrain water intake [18–21]. Sodium pentobarbital (75 mg/kg) was injected into the abdomen for anesthesia. Fixed in supine position, II lead electrocardiogram was recorded. The skin and trachea of the neck and chest surgical site were cut open and exposed. The animal ventilator was connected (respiration rate 70 times/min, suction/breath ratio 1 : 2, and tidal volume 9 ml/kg). Cut the skin from the 3^rd^ to 4^th^ intercostals on the left. Strip muscle tissue. Open the chest and cut the capsule. Locate the left anterior descending coronary artery between the left auricle and pulmonary conus and ligate with 5-0 wire about 1 mm outside the starting point of the branch. At the same time, ECG was recorded. The ST segment of the lead II of standard limb was lifted up with *T* wave soaring, indicating myocardial ischemia. The reperfusion model was loosened after ligation for 30 min to induce the reperfusion of the ischemic coronary artery. Thoracic reperfusion was closed for 120 minutes. ECG showed that ST segment dropped more than 1/2, indicating that the modeling was successful. Death because of abnormal electrocardiogram or failure to reach the observation end point before ligation and unsuccessful modeling were eliminated. The sham operation group did not ligate the coronary arteries after thoracotomy but only used a needle to puncture the corresponding site once. The rats were euthanized with carbon dioxide. Place the animal in a clean container and slowly inject carbon dioxide. Ten minutes later, the rats were euthanized. Wait another 2 minutes and check whether the rats were dead one by one. If undead animals are found, cervical vertebra dislocations are supplemented. All animal operation procedures are in accordance with the ethical review of animal experiments and also meet the ethical requirements of animal welfare. This study was approved by the animal ethics committee of Putuo Hospital (No. 20190232).

The article "Therapeutic Effect and Mechanism of Cinnamyl Alcohol on Myocardial Ischemia-Reperfusion Injury" was retracted in 2023. Reasons: signs of a paper mill; compromised peer review; unreliable results or conclusions.

### 2.2. HE

The heart was extracted and cleaned with PBS. The cardiac tissue (>1 mm^3^) was taken from the apex of the heart, and it was decalcified, dehydrated, transparent, and waxed. The biological tissue embedding machine was used for embedding. The LEICARM2016 tissue slicer was used. Hematoxylin was dyed for 5 min. After rinsing with water for 5 minutes, 1% hydrochloric acid ethanol was used for 30 seconds. Wash with distilled water for 5 s and dye with 0.5% eosin solution for 1–3 min. Rinse with distilled water for 30 seconds. After HE staining, observe and take pictures under an optical microscope.

### 2.3. Cell Culture

Place the H9c2 cardiomyocyte cell line in a 37°C, 95% air, 5% CO_2_ incubator. Culture with DMEM complete medium containing 15% fetal bovine serum. When the cell fusion degree is about 85%, perform trypsin digestion with a mass concentration of 0.25 g/L. Count and inoculate 1.0 × 10^6^ cells in a 25 cm^2^ culture flask for passage. The fluid was changed every 2 d, and the cells were passaged every 3–4 d. The cardiomyocytes in the logarithmic growth phase were used for subsequent experiments.

The article "Therapeutic Effect and Mechanism of Cinnamyl Alcohol on Myocardial Ischemia-Reperfusion Injury" was retracted in 2023. Reasons: signs of a paper mill; compromised peer review; unreliable results or conclusions.

### 2.4. Cell Hypoxia/Reoxygenation Model

After the cells have reached 95% fusion, discard the cell culture medium. Add serum-free DMEM simulated hypoxia solution saturated with the mixed gas of 37°C, 95% N_2_, and 5% CO_2_ for 30 minutes. Put it into the hypoxic chamber, and pass in a mixture of 95% N_2_ and 5% CO_2_ for 5 minutes to drive off oxygen. Place it in a 37°C incubator for 21 h to conduct hypoxia. Then, replace the hypoxic fluid with a normal medium. Incubate in a 37°C, 95% air, and 5% CO_2_ incubator for 6 hours to simulate reoxygenation.

### 2.5. Cell Transfection

ATG12 siRNA and negative control siRNA were transfected into cardiomyocytes by Lipofectamine™ 2000. Dilute an appropriate amount of Lipofectamine™ 2000 and ATG 12siRNA with serum-free DMEM medium according to the operating instructions to form a transfection reagent mixture. Add to a 6-well plate with a 90% cardiomyocyte density. Shake gently to mix. After culturing in a 5% CO_2_ incubator for 6 hours, the culture medium was replaced with serum. After 48 hours of transfection, transfection efficiency verification and follow-up experiments were carried out.

### 2.6. qRT-PCR

The myocardial tissue was homogenized to extract RNA. Use the rapid reverse transcription kit to synthesize the first strand cDNA. 2 *μ*g total RNA was used to establish a 20 *μ*L reaction system. Incubate at 42°C for 15 minutes and at 95°C for 3 minutes, then place on ice. The obtained cDNA can be used in real-time PCR reaction. Use a real-time quantitative PCR machine to set up the reaction program. Perform PCR amplification and read the data. GAPDH upstream: GTTACCAGGGCTGCCTTCTC; downstream: GATGGTGATGGGTTTCCCGT. ATG12, Forward: 5′-CTGCTGCGGCGGGCGAGAG-3′; Reverse: 5′-GGGCGAAACTGCAACCGAAGACG-3′. The amplification procedure is as follows: perform denaturation at 95°C for 5 min, and then perform 40 cycles of denaturation at 94°C for 20 s and annealing at 60°C for 20 s. Obtain the cycle threshold (Ct) of mRNA. The ^△△^Ct (^△△^Ct = ^△^Ct target gene ^−△^Ct internal reference gene) method was used to analyze, and after calculating the relative expression of 2^−△△Ct^ target gene, statistical analysis was performed. The qRT-PCR experiment was repeated three times.

### 2.7. Western Blot

The rat myocardial tissue was homogenized and centrifuged. Cell lysis conditions were as follows: RIPA lysate (strong) + 100 *μ*M PMSF(100×) + Cocktail (100×). Take the supernatant and use the BCA method to determine the protein concentration. The cardiomyocytes are treated with lysate. Take 30 *μ*g samples of each group for 10% SDS-PAGE. The protein sample is transferred to the PVDF membrane. The skimmed milk powder was blocked for 1 hour at room temperature to block nonspecific antigens. The primary antibody was diluted 1 : 1000 with 5% BSA-TBST. Incubate overnight at 4°C. Then, dilute the HRP secondary antibody at a ratio of 1 : 1000. Incubate at room temperature for 40 minutes. Add an appropriate amount of luminescent substrate reagent to each film to perform chemiluminescence and obtain the result. The positive bands were analyzed with Gelpro 4.0 version gel optical density software, and the integrated optical density (IOD) was measured.

The article "Therapeutic Effect and Mechanism of Cinnamyl Alcohol on Myocardial Ischemia-Reperfusion Injury" was retracted in 2023. Reasons: signs of a paper mill; compromised peer review; unreliable results or conclusions.

### 2.8. Cell Proliferation Detection

Take the growth phase cells and inoculate 5000 cells per well in a 96-well plate. Ensure regular cultivation for 24 h. After transfection or treatment with CA for 48 hours, add 10 *μ*L of CCK-8 solution to each well. Incubate at 37°C for 1 h. Detect the absorbance (*A*) value of each well at 450 nm wavelength with a microplate reader.

### 2.9. TUNEL

4% paraformaldehyde was fixed at 4°C for 30 min. Wash with PBS 3 times, 5 min each time. Punch holes for 10 minutes at room temperature with 0.3% Triton X-100. Wash with PBS 3 times, 5 min each time. Strictly follow the instructions of the TUNEL kit (one-step TUNEL cell apoptosis detection kit, C1088, Beyotime, Shanghai, China), and mix the No. 1 and No. 2 solutions in the ratio of 1 : 9 in the dark. The mixed solution was dropped on the cells. Incubate for 1 h in a 37°C water bath protected from light. Wash with PBS 3 times, 5 min each time. The nuclei were counterstained with DAPI and incubated in a 37°C water bath protected from light for 10 minutes. Wash with PBS 3 times, 5 min each time. The results of TUNEL staining were photographed by fluorescence microscope (Nikon, Japan). The percentage (%) of the cell nucleus using green fluorescence in the total cell nucleus represents the apoptosis rate (apoptotic index).

### 2.10. Statistical Analysis

GraphPad Prism 5.0 statistical software was used for data analysis. The data of each group are expressed as mean ± SD. The unpaired Student's *t*-test was used for comparison between the two groups. The one-way analysis of variance (one-way ANOVA) was used for the comparison of means between multiple groups, and the Tukey test was used for multiple comparisons. The difference was statistically significant when *P* < 0.05.

## 3. Results

### 3.1. CA Inhibits Inflammation after Myocardial Infarction and Protects the Myocardial Tissue

To study the myocardial protective effect of CA, an animal model of myocardial ischemia-reperfusion injury was first established. It can be seen from Figure 1(a) that the myocardial tissue structure of the rats in the sham operation group is clear, the myocardial fibers are arranged neatly, the structure is complete, the myocardial fibers are rarely broken, and there is no interstitial edema of myocardial cells. In the model group, the arrangement of the myocardial tissue was disordered, myocardial fibers were extensively degenerated and broken, and the interstitium of the myocardial cells was edema. The myocardial tissues of the rats in the CA treatment group were arranged neatly, no myocardial fibers were broken, and the interstitium of the myocardial cells slightly had edema. qRT-PCR was used to detect the mRNA expression of IL-1*β*, IL-6, and TNF*α* in the myocardial tissue. The results showed that compared with the sham operation group, the expression of IL-1*β*, IL-6, and TNF*α* in the model group was significantly increased (*P* < 0.01), indicating that myocardial ischemia reperfusion can induce cellular inflammation. In the CA administration group, the expression of IL-1*β*, IL-6, and TNF*α* decreased, which was significantly different from the model group (*P* < 0.01). It shows that CA can inhibit myocardial ischemia-reperfusion and induce cellular inflammation (Figures 1(b)–1(d)). TUNEL was used to detect the degree of apoptosis of cardiomyocytes. As shown in Figure 1(e), compared with the sham operation group, the apoptosis of the myocardial tissue in the model group increased, indicating that the myocardial ischemia-reperfusion injury model was successfully established. After the intervention of CA, compared with the model group, the degree of myocardial cell apoptosis showed a downward trend (*P* < 0.01), indicating that CA can reduce myocardial cell damage caused by myocardial ischemia and reperfusion. The qRT-PCR results showed that compared with the sham operation group, the expression of pro-apoptotic proteins Bax and Cyt-c in the model group increased significantly (*P* < 0.01). Compared with the model group, CA treatment can significantly downregulate the expression levels of Bax and Cyt-c (Figures 1(f)-1(g), *P* < 0.01). qRT-PCR was used to detect the mRNA expression of Bcl-2 in the myocardial tissue. The results showed that CA treatment can upregulate the expression of the antiapoptotic gene Bcl-2 (Figure 1(h)).

The article "Therapeutic Effect and Mechanism of Cinnamyl Alcohol on Myocardial Ischemia-Reperfusion Injury" was retracted in 2023. Reasons: signs of a paper mill; compromised peer review; unreliable results or conclusions.

### 3.2. CA Reduces Autophagy and Inhibits Myocardial Ischemia-Reperfusion Injury

Subsequently, we detected changes in the expression of autophagy-related proteins. Compared with the sham operation group, the expression of Beclin-1, P62 protein, and the ratio of LC3 II/LC3 I in the model group increased, indicating that myocardial ischemia reperfusion can induce autophagy. Compared with the model group, CA treatment can significantly downregulate the expression of Beclin-1, p62 protein, and the ratio of LC3 II/LC3 I (*P* < 0.01). It shows that CA can inhibit myocardial ischemia-reperfusion and induce autophagy (Figure 2).

### 3.3. CA Inhibits the Autophagy Response of Cardiomyocytes Caused by Hypoxia-Reperfusion Injury

Through hypoxia/reoxygenation treatment of cardiomyocytes, an *in vitro* myocardial ischemia-reperfusion injury cell model was constructed. To further evaluate the protective effect of CA on cardiomyocytes. qRT-PCR was used to detect the mRNA expression of IL-1*β*, IL-6, and TNF*α* in the cardiomyocytes. The results showed that, compared with the control group, the expression of IL-1*β*, IL-6, and TNF*α* in the hypoxia/reoxygenation model group increased significantly (*P* < 0.01). In the CA administration group, the expression of IL-1*β*, IL-6, and TNF*α* decreased, which was significantly different from the model group (*P* < 0.01). It shows that CA can inhibit myocardial ischemia-reperfusion and induce cellular inflammation (Figures 3(a)–3(c)). Western blot detection of Beclin1, p62, LC3-I, and LC3-II expression changes in different treatment groups showed that, compared with the control group, the H/R model group Beclin-1, P62 protein expression, and LC3 II/LC3 I ratio increased. Compared with the H/R model group, CA treatment can significantly downregulate the expression of Beclin-1, p62 protein, and the ratio of LC3 II/LC3 I (*P* < 0.01). It shows that CA can inhibit autophagy caused by hypoxia/reoxygenation treatment (Figures 2(d)–2(g)).

### 3.4. CA Targets ATG12

Autophagy-related protein 12 (ATG12) is a ubiquitin-like protein involved in the formation of autophagy vesicles. ATG12 can participate in the autophagy and apoptosis-related processes of cells and the damage repair process of tissues and organs by regulating the formation of autophagy complexes.  Figure 4(a) experimental results show that the expression of ATG12 is upregulated in the animal models of myocardial ischemia-reperfusion injury. After treatment with CA, the expression of ATG12 in the rat myocardial tissue decreased (Figure 4(b)). In addition, in cardiomyocytes, the expression of ATG12 was upregulated after H/R induction treatment (Figure 4(c)). In cardiomyocytes, after CA intervention, the expression of ATG12 decreased compared with the model group (Figure 4(d)). It shows that CA inhibits the upregulation of ATG12 expression induced by H/R.

### 3.5. Knockdown of ATG12 Reduces the Production of Inflammatory Cytokines Triggered by H/R

Compared with the si-NC group, after si-ATG12 transfection, the expression of ATG12 in the cardiomyocytes decreased (Figure 5(a)). qRT-PCR was used to detect the mRNA expression of IL-1*β*, IL-6, and TNF*α* in the cardiomyocytes. The results showed that under the background of hypoxia/reoxygenation induction treatment, compared with the control group, knocking down ATG12 can reduce the expression of IL-1*β*, IL-6, and TNF*α*. Experimental results show that knocking down ATG12 reduces H/R-induced increase in cytoinflammatory factors in the supernatant of cardiomyocytes.

The article "Therapeutic Effect and Mechanism of Cinnamyl Alcohol on Myocardial Ischemia-Reperfusion Injury" was retracted in 2023. Reasons: signs of a paper mill; compromised peer review; unreliable results or conclusions.

### 3.6. Knockdown ATG12 Inhibits H/R-Mediated Cardiomyocyte Damage

The results of cell proliferation experiments showed that compared with the normal control group, H/R treatment inhibited the cell proliferation ability. Compared with the H/R model group, knocking down ATG12 or treating with CA can restore the proliferation ability of the cardiomyocytes (Figure 6(a)). The results of the TUNEL experiment showed that compared with the normal control group, H/R treatment promoted cardiomyocyte apoptosis. Compared with the H/R model group, the knockdown of ATG12 or CA treatment can reduce the level of cardiomyocyte apoptosis (Figure 6(b)). The results of qRT-PCR showed that, compared with the normal control group, the expression of proapoptotic genes Bax and Cyt-c increased significantly in the H/R model group. Compared with the H/R model group, the knockdown of ATG12 or CA treatment can reduce the expression levels of Bax and Cyt-c (Figures 6(c)-6(d)). qRT-PCR was used to detect the mRNA expression of Bcl-2 in the cardiomyocytes. The results showed that the expression of Bcl-2 decreased after H/R treatment. The knockdown of ATG12 or CA treatment can upregulate the expression of the antiapoptotic gene Bcl-2 (Figure 6(e)).

## 4. Discussion

Studies have shown that the pathogenesis of myocardial ischemia-reperfusion injury mainly includes energy metabolism disorder, excessive ROS production, calcium overload, inflammatory response, apoptosis, and autophagy [22]. Autophagy plays an important role in maintaining homeostasis, resisting environmental changes, stress, and inflammatory responses [23]. When autophagy is overexpressed or the stress and inflammatory response are strong, the protective effect of autophagy will be transformed into autophagy cell death or apoptosis [24]. Myocardial ischemia is essentially a nutrient deficiency caused by inadequate blood flow. Therefore, autophagy can be induced by ischemia [25]. Moreover, the reperfusion process promotes the formation of autophagosomes. In the stage of cardiac reperfusion, oxidative stress, mitochondrial injury and inflammatory reaction can cause the excessive activation of autophagy, resulting in the excessive degradation of important proteins and organelles, and it ultimately induces irreversible cell death. Beclin-1 is a key gene that regulates autophagy. Beclin-1 expression level reflects autophagy activity to a certain extent. LC3 is a signature protein of autophagy, which is divided into two subtypes [26]. During autophagy, LC3 I is clipped to form LC3 II. LC3 II plays an important role in autophagic vesicle formation. Therefore, LC3 II/LC3 I ratio can reflect the degree of autophagy activation under stress [27]. In this study, protein levels of Beclin-1, P62, LC3 II, and LC3 II/LC3 I significantly increased after reperfusion, indicating that autophagy was activated and overexpression level was maintained. Further experimental results showed that CA could inhibit autophagy.

The article "Therapeutic Effect and Mechanism of Cinnamyl Alcohol on Myocardial Ischemia-Reperfusion Injury" was retracted in 2023. Reasons: signs of a paper mill; compromised peer review; unreliable results or conclusions.

Understanding the molecular mechanism of myocardial cell apoptosis during myocardial ischemia-reperfusion injury and conducting in-depth research on the important targets and pathways of myocardial cell apoptosis is of great significance for alleviating the injury caused by hypoxia and ischemia [28]. The formation of autophagosomes includes the binding process of ATG12 and the modification process of LC3 [29]. ATG12 is activated by Atg7 and is transferred to Atg10, and finally, it binds with Atg5 to form the autophagic progenitor. Soluble LC3 I was formed in the cytoplasm after the processing of the LC3 precursor. LC3 I is also transported to Atg3 by Atg7, where it is modified and processed to form LC3 II [30, 31]. LC3 II is a marker factor of autophagy, and its content can determine the autophagy state of cells [32]. The role of ATG12 in regulating apoptosis is very complex. ATG12 has both antiapoptotic and proapoptotic effects [33]. Studies have shown that ATG12 is involved in inducing apoptosis, and the protein inhibits the activity of antiapoptotic proteins and promotes apoptosis by interacting with antiapoptotic members of the Bcl-2 family [34].

Many Traditional Chinese medicines can regulate autophagy [15, 35–37]. For example, Sal B, derived from *Salvia miltiorrhiza*, inhibits autophagy at the early stage of autophagy by blocking the autophagy flow and affecting the formation of autophagosomes, and it alleviates cell apoptosis during autophagy [38]. Recent studies have shown that Sal B can inhibit autophagy by downregulating the expression of Beclin-1 and LC3-II. However, Sal B-induced p-Akt expression and antiautophagy effect were eliminated with PI3K inhibitor LY294002. Therefore, Sal B's inhibition of autophagy may reduce myocardial cell I/R injury by regulating the PI3K/Akt signaling pathway [39]. Total flavonoid (BCF) is the main active component of the stem extract of *Pterygium spinosa*. Studies have shown that BCF can scavenge free radicals, improve myocardial energy metabolism, and reduce inflammatory responses and myocardial damage. BCF inhibits apoptosis and promotes the survival rate of cardiomyocytes damaged by hypoxia/reoxygenation [40]. BCF preconditioning downregulated beclin-1 and LC3-II, upregulated PI3K and p-Akt protein expressions, and increased endothelial nitric oxide synthase (eNOS) protein levels [41].

The article "Therapeutic Effect and Mechanism of Cinnamyl Alcohol on Myocardial Ischemia-Reperfusion Injury" was retracted in 2023. Reasons: signs of a paper mill; compromised peer review; unreliable results or conclusions.

In this study, it was found that CA inhibited ATG12 and downregulated LC3 and Beclin-1 gene expression, which inhibit autophagy in MI/RI. CA reduced mitochondrial peroxidation and improved myocardial cell apoptosis. The result was increased myocardial protection in MIRI rats. It may be one of the mechanisms of the effect of CA on myocardial protection.

## 5. Conclusion

Autophagy plays an important role in ischemia-reperfusion injury. The change of autophagy is directly related to the survival of cardiac myocytes. The results showed that after MI/RI, the expression level of ATG12 increased, autophagy expression was rapidly upregulated, and myocardial apoptosis was serious. CA can inhibit the autophagy of cardiomyocytes by inhibiting ATG12 and reduce apoptosis response, thus playing a protective role in myocardial ischemia-reperfusion injury.

## Figures and Tables

**Figure 1:** CA inhibits inflammation after myocardial infarction and protects myocardial tissue. (a) HE staining to evaluate the damage of the myocardial tissue. (b) qRT-PCR detects the mRNA expression of IL-1*β* in the myocardial tissue. (c) qRT-PCR detects the mRNA expression of IL-6 in the myocardial tissue. (d) qRT-PCR detects the mRNA expression of TNF*α* in the myocardial tissue. (e) The myocardial tissue TUNEL detects the degree of apoptosis. (f) qRT-PCR detects the mRNA expression of Bax in the myocardial tissue. (g) qRT-PCR detection of Cyt-c mRNA expression in the myocardial tissue. (h) qRT-PCR detects the mRNA expression of Bcl-2 in the myocardial tissue. Data are presented as the mean ± SD. ^*∗*^*P* < 0.05 and ^*∗∗*^*P* < 0.001.

**Figure 2:** CA reduces autophagy and inhibits myocardial ischemia-reperfusion injury. (a) Western blot detection of Beclin1, p62, LC3-I, and LC3-II expression changes in different treatment groups. (b) Beclin expression statistics results. (c) Statistical results of p62 expression. (d) Statistical results of LC3-I and LC3-II expression changes. Data are presented as the mean ± SD. ^*∗*^*P* < 0.05 and ^*∗∗*^*P* < 0.001.

**Figure 3:** CA inhibits the autophagy response of cardiomyocytes caused by hypoxia-reperfusion injury. (a) qRT-PCR detects the mRNA expression of IL-1*β* in the myocardial tissue. (b) qRT-PCR detects the mRNA expression of IL-6 in the myocardial tissue. (c) qRT-PCR detects the mRNA expression of TNF*α* in the myocardial tissue. (d) Western blot detection of Beclin1, p62, LC3-I, and LC3-II expression changes in different treatment groups. (e) Beclin expression statistics results. (f) Statistical results of p62 expression. (g) Statistical results of LC3-I and LC3-II expression changes. Data are presented as the mean ± SD. ^*∗*^*P* < 0.05 and ^*∗∗*^*P* < 0.001.

The article "Therapeutic Effect and Mechanism of Cinnamyl Alcohol on Myocardial Ischemia-Reperfusion Injury" was retracted in 2023. Reasons: signs of a paper mill; compromised peer review; unreliable results or conclusions.

**Figure 4:** CA targets ATG12. (a) The expression of ATG12 is upregulated during myocardial ischemia. (b) CA inhibits the expression of ATG12. (c) In cardiomyocytes, H/R induces the upregulation of ATG12 expression. (d) In cardiomyocytes, CA inhibits the upregulation of ATG12 expression induced by H/R. Data are presented as the mean ± SD. ^*∗∗*^*P* < 0.001.

**Figure 5:** Knockdown of ATG12 reduces the production of inflammatory cytokines triggered by H/R. (a) Verification of siRNA ATG12 knockdown efficiency. (b) IL-1*β* expression detection. (c) IL-6 expression detection. (d) TNF*α* expression detection. Data are presented as the mean ± SD. ^*∗*^*P* < 0.05 and ^*∗∗*^*P* < 0.001.

**Figure 6:** Knockdown of ATG12 inhibits H/R-mediated cardiomyocyte damage. (a) Detection of cardiomyocyte proliferation. (b) TUNEL detects cell apoptosis. (c) qRT-PCR detects the mRNA expression of Bax in cardiomyocytes. (d) qRT-PCR detection of Cyt-c mRNA expression in cardiomyocytes. (e) qRT-PCR detection of Bcl-2 mRNA expression in cardiomyocytes. Data are presented as the mean ± SD. ^*∗*^*P* < 0.05 and ^*∗∗*^*P* < 0.001.

## Data Availability

The data used to support the findings of this study are available from the corresponding author upon request.
